The article "Metaheuristic-based Deep COVID-19 Screening Model from Chest X-Ray Images" was published in 2021. Journal: J Healthc Eng.

# Metaheuristic-based Deep COVID-19 Screening Model from Chest X-Ray Images

**DOI:** 10.1155/2021/8829829

**Published:** 2021-03-01

**Authors:** Manjit Kaur, Vijay Kumar, Vaishali Yadav, Dilbag Singh, Naresh Kumar, Nripendra Narayan Das

**Affiliations:** ^1^Computer Science Engineering, School of Engineering and Applied Sciences, Bennett University, Greater Noida, 201310, India; ^2^Department of Computer Science and Engineering, National Institute of Technology Hamirpur, Hamirpur, Himachal Pradesh, 177005, India; ^3^Department of Computer and Communication Engineering, School of Computing and Information Technology, Manipal University Jaipur, Jaipur, Rajasthan, 303007, India; ^4^Department of Computer Science and Engineering, Maharaja Surajmal Institute of Technology, C-4 Block, Janakpuri, New Delhi 110058, India; ^5^Department of Information Technology, School of Computing and Information Technology, Manipal University Jaipur, Jaipur, Rajasthan, 303007, India

## Abstract

COVID-19 has affected the whole world drastically. A huge number of people have lost their lives due to this pandemic. Early detection of COVID-19 infection is helpful for treatment and quarantine. Therefore, many researchers have designed a deep learning model for the early diagnosis of COVID-19-infected patients. However, deep learning models suffer from overfitting and hyperparameter-tuning issues. To overcome these issues, in this paper, a metaheuristic-based deep COVID-19 screening model is proposed for X-ray images. The modified AlexNet architecture is used for feature extraction and classification of the input images. Strength Pareto evolutionary algorithm-II (SPEA-II) is used to tune the hyperparameters of modified AlexNet. The proposed model is tested on a four-class (i.e., COVID-19, tuberculosis, pneumonia, or healthy) dataset. Finally, the comparisons are drawn among the existing and the proposed models.

## 1. Introduction

Severe acute respiratory syndrome coronavirus 2 (SARS-CoV-2) causes this disease. Several other viruses like MERS, flu, and SARS [1–3] have also been detected in the past few decades, but they have not affected the world as COVID-19 does. Many countries are working on preparing a vaccine to get over this pandemic. Since this is an infectious disease and appropriate treatment is not available to date, it is highly required that the disease is detected in the early stages so that its further spreading can be prevented [4]. The symptoms of COVID-19 are sore throat, fever, headache, breathing issues, and cough [5]. Some other symptoms like tiredness, aches, loss of taste, and smell have also been found in some patients. However, in many of the infected patients, no symptoms were reported [6]. Because of the absence of symptoms, it became much difficult to detect the COVID-19 infection. Hence, many countries declared lockdown so that the chain of the disease can be broken. But still, for treating the disease, efficient screening of patients is needed.

The article "Metaheuristic-based Deep COVID-19 Screening Model from Chest X-Ray Images" was published in 2021. Journal: J Healthc Eng.

Real-time reverse transcription-polymerase chain reaction (RT-PCR) is widely accepted as a COVID-19 detection tool [7]. It can provide results ranging from hours to two days. But, because of the unavailability of kits and RT-PCR's low sensitivity, the imaging techniques utilizing radiography emerged as another option for COVID-19 detection [8]. Several research articles also validate the suitability of chest scans for the detection of COVID-19 [7, 8]. Among available radiography techniques, the chest CT scan and X-ray are extensively utilized techniques. But the availability of machines and lesser impact of radiations on patients make X-rays more preferable over CT [9]. It takes much time and can lead to erroneous reports when the X-rays are examined manually by radiological experts [10]. This problem can be resolved by analyzing the X-ray automatically by using the machine/deep learning models. In recent times, deep learning techniques have been favorites among researchers to diagnose diseases in the field of medical imaging [11]. These techniques can extract the image features automatically without any manual involvement [12] which makes them suitable for the classification process of COVID-19 imaging patterns.

This paper proposes a metaheuristic-based deep COVID-19 screening model for X-ray images. The modified AlexNet architecture is used for feature extraction and classification of the input images. Strength Pareto evolutionary algorithm-II (SPEA-II) is used to tune the hyperparameters of modified AlexNet. The proposed model is tested in a four-class (i.e., COVID-19, tuberculosis, pneumonia, or healthy) dataset. Finally, the comparisons are drawn among the existing and the proposed models.

The remaining structure of the paper is as follows.  Section 2 describes the related work in the field. The proposed work for detecting COVID-19 using chest X-rays is presented in Section 3.  Section 4 discusses the experimental results and discussions. The proposed work is concluded in Section 5.

## 2. Literature Review

In the last few months, several deep learning techniques have been rigorously used for the classification of chest X-rays for COVID-19 diagnosis. Among these techniques, convolutional neural networks (CNNs) and transfer learning have been explored a lot. Hemdan et al. [13] proposed an automatic framework named “COVIDX-Net” to identify the COVID-19 infection in chest X-rays. The proposed model used seven deep learning architectures, out of which DenseNet201 and VGG19 achieved 90% accuracy. The authors used only fifty chest X-rays to test the proposed model. In [14], deep learning architectures are studied by Luz et al., and the efficiency of the proposed model is presented using the COVIDx dataset. The accuracy of 93.9% with 96.8% sensitivity is achieved by the Flat EfficientNet model. Ozturk et al. [15] developed DarkCovidNet, an automatic model for detecting COVID-19 using chest X-rays. The model is trained using 125 chest images and provided 98.08% accuracy with binary cases and 87.02% accuracy with multiclass cases. The use of a limited number of COVID-19-infected chest X-ray images for training and validation purposes is the main drawback of this model. Basu and Mitra [16] proposed a model for identifying abnormality caused by COVID-19 in chest X-rays. This model is based on transfer learning; they used Gradient Class Activation Map for extracting features from X-ray images. Validation is also done with the help of the NIH chest X-ray dataset. Results achieved are also promising with an overall accuracy of 95.3%. Das et al. [17] proposed a model for the detection of COVID-19 infection with the help of X-ray images. In this work, the developed model is based on the deep learning technique. The experimental results show an overall classification accuracy of 97.40%.

The article "Metaheuristic-based Deep COVID-19 Screening Model from Chest X-Ray Images" was published in 2021. Journal: J Healthc Eng.

Tuncer et al. [18] proposed a model to identify the COVID-19 pattern from the X-ray images. In this, features are extracted with Residual Exemplar Local Binary Pattern (ResExLBP). Feature selection is done with iterative ReliefF. In this work, a total of 321 chest X-ray images are used to achieve the classification accuracy of 99% with an SVM classifier. Wang and Wong [19] implemented a COVID-Net framework for identifying coronavirus infection. The proposed framework reports the classification accuracy as 92.4% for normal, pneumonia+ve, and COVID+ve classes, which are better than VGG19 and ResNet-50 architecture. Toğaçar et al. [20] converted the original X-rays of COVID-19 patients into a useful structured dataset with the help of fuzzy color technique; then, an image stacking technique has been used to create a stacked dataset. In this, the classification accuracy of MobileNetV2 and SqueezeNet is 98.25% and 97.81%, respectively.

Apostolopoulos and Mpesiana [21] proposed a COVID-19 identification system. In this work, five pretrained deep learning architectures were used to develop the system for the processing of chest X-ray images. VGG19, MobileNet, Inception, Xception, and Inception_ResNet_V2 are the pretrained deep learning architectures. Classification accuracy is also very good for a binary class as compared with multiclass. Mahmud et al. [22] developed an automatic system CovXNet for COVID-19. The proposed system detects the COVID-19 patterns from chest X-rays. A total of 915 X-ray images were used to validate the model. The proposed system is optimized with the help of a stacking algorithm. Classification is also done with binary and three classes with an accuracy of 97.4% and 89.6%, respectively. In Narin et al. [23], the work performance of three pretrained deep learning architectures is analyzed for COVID-19. ResNet50, Inception_V3, and Inception-ResNet_V2 were executed and concluded that ResNet50 is the best among all with 98% accuracy. Shelke et al. [24] proposed a diagnosis model for COVID-19 based on chest X-ray images. In this work, 22 X-ray images were used to calculate the classification accuracy and it is 98.9%.

The article "Metaheuristic-based Deep COVID-19 Screening Model from Chest X-Ray Images" was published in 2021. Journal: J Healthc Eng.

Rahimzadeh and Attar [25] proposed a hybridized model for COVID-19 by combining Xception and ResNet50_V2 models. A dataset of 6054 X-ray images was used, and 91.4% accuracy has been achieved. In Chouhan et al. [26], an ensemble approach has been proposed for AlexNet, DenseNet121, Inception_V3, ResNet18, and GoogleNet architectures. These pretrained deep learning architectures show good accuracy for COVID-19 pattern identification. Abbas et al. [27] developed a DeTraC model for predicting COVID-19 with the help of 105 chest X-ray images. CNN model has been used for deep feature extraction. Also, class decomposition is implemented to extract the local structures. 95.12% classification accuracy is achieved with Gradient descent. Das et al. [28] used an open-source chest X-ray dataset for the identification of COVID-19. A model is implemented using the InceptionNet model and achieved promising results. From the above literature, it has been found that the existing model suffers from the overfitting and hyperparameter-tuning issue [29].

## 3. Proposed Methodology

This section discusses the proposed work. CNN is discussed followed by modified AlexNet architecture and SPEA-II-based hyperparameter- tuning approach.

### 3.1. Convolutional Neural Network (CNN)

CNN emulates the human brain's functioning. The layers in CNN work like layers of the human brain. It can be termed as a deep learning neural network [30, 31]. CNN has proven its efficacy in pattern recognition, face recognition, and other image processing applications. Different layers in the CNN process the input image [32]. In the initial convolution layer, the input image is fed; then, different layers of the proposed architecture extract the features. In the convolutional layer, the input image goes through different filters; then, the output of this layer is passed as input to the next layer called the maximum pooling layer which removes the unwanted pixels [33].

The article "Metaheuristic-based Deep COVID-19 Screening Model from Chest X-Ray Images" was published in 2021. Journal: J Healthc Eng.

In this paper, AlexNet architecture is used for CNN because it is computationally better to use the AlexNet architecture to address the complexities than Conv-Net, Le-Net, ResNet, and other architectures [27]. Initially, a set of images are assigned to the first layer of AlexNet. Hidden layers apply multiple filters to extract the features. Finally, the last layer is used for the classification process [34].

### 3.2. AlexNet Architecture

As stated earlier, AlexNet is better than the other available architectures in terms of efficiency and computational ability. These are also used extensively to cope up with the problems in the process of image classification. This paper uses the modified AlexNet architecture [35] for image classification.  Figure 1 shows the detailed architecture used for image classification.

The implementation of the modified architecture is comprised of the following steps:

  Step 1: initially, the input image is resized to 259 × 259 pixels representing the length and breadth. The depth is represented by three color channels.
  Step 2: next operation carried out in the convolutional layer computed the output of neurons by performing the scalar product of the image's small portions with their respective weights. This operation is iterated along length and breadth.
  Step 3: then, the ReLU layer employs an activation function that works element-wise. It also incorporates the nonlinearity in the system and applies the function due to which the negative activation is replaced by 0.
  Step 4: the decimation operation is performed at the pooling layer which reduces the samples along with the spatial coordinates.
  Step 5: at last, the prediction is given by a fully connected (FC) layer based on a class score of each image. For each prediction class, the probability score is computed and the class with the maximum probability score is considered to be the predicted class.

### 3.3. Strength Pareto Evolutionary Algorithm (SPEA)

To optimize CNN, SPEA-II [36] is used in this work. The idea of SPEA [37] was introduced in 1999. But to understand SPEA-II, we need to understand the working of SPEA. In SPEA, Strength Pareto depicts how much the solutions are close to the first rank. The nondominated solutions or a set of Pareto optimal solutions are identified and preserved with SPEA. A set containing all Pareto optimal solutions is called Pareto optimal set, and it contains the best nondominated solutions. For each solution, two parameters named Strength Pareto (*S*) and fitness (*F*) are considered. The Strength Pareto is represented as

(1) $$\begin{array}{c} S\left(i\right)=\frac{\text{np}}{\text{NP}+1}, \end{array}$$

where *S*(*i*) represents the Strength Pareto of individual *i*. NP represents the size of the population and np is the number of individual vectors that are dominated by individual *i* or having equal strength as *i*. These dominated individuals possess less strength than the nondominated solutions. The second parameter, i.e., fitness, is represented as [38]

(2) $$\begin{array}{c} F\left(a\right)=1+\sum_{i<a}S\left(i\right). \end{array}$$

The fitness of an individual *a* is the addition of Strength Pareto values of all individuals which dominate or equal individual *a*. Hence, the solution with a lower value of fitness is assumed to be better [38]. Consider *G* as the maximum number of generations and *g* as the iteration number. The steps involved in the optimization process of SPEA are described as follows.

  Step 1: the population is initialized and an empty external set is created for Pareto optimal solutions.
  Step 2: the size of Pareto optimal is defined; if it exceeds that limit, then based on the average linkage-based hierarchical clustering method, Pareto sets are deleted and brought back to a manageable size. This clustering technique combines the adjacent clusters iteratively until the desired number of groups is obtained [38].
  Step 3: next, the fitness of the population and external Pareto optimal set is calculated [39].
  Step 4: in this step, binary tournament selection is implemented by combining the individuals in an external set and the population. Then, two individuals are chosen randomly and one having better fitness is moved to the mating pool. In the mating pool, crossover operation and mutation operations are performed so that a new population is obtained for the next iteration.
  Step 5: a new population is assumed to have better individuals than the previous one generated by perturbation and crossover.
  Step 6: increase *g* as *g*=*g*+1 and check for the termination condition. If the termination condition is not satisfied, then go to Step 2; else, represent the archive members as Pareto optimal set [39].

The article "Metaheuristic-based Deep COVID-19 Screening Model from Chest X-Ray Images" was published in 2021. Journal: J Healthc Eng.

### 3.4. SPEA-II

Figure 2 shows the *i*^*th*^ generation of SPEA-II. Having *T*_*g*_ (as the population at *g*^*th*^ iteration), $\bar{T_{g}}$ (as the archive population at *g*^*th*^ iteration), *G* (as the max number of generations), and $\bar{A}$ as archive size, the steps of the optimization process followed by SPEA-II are as follows [36].

  Step 1 (initialization): initialize an empty archive $\bar{T_{g}}=\varphi$ and an initial population *T*_0_ and set *g* = 0.
  Step 2 (fitness calculation): in this step, the fitness of the population and the archive set individuals are calculated. The strength *S(i)* of individual *i* in population and the archive is calculated as
  (3) $$\begin{array}{c} S\left(i\right)=\left|\left\{a|a\in T_{g}+{\bar{T}}_{g}\wedge i>a\right\}\right|. \end{array}$$
Here, “+” represents the multiset union, “∧” represents the AND operation, and “>” represents the Pareto dominance relation.
Fitness *F*(*i*) for SPEA-II is calculated using raw fitness *P*(*i*) and density *Q*(*i*) of an individual as
  (4) $$\begin{array}{c} F\left(i\right)=P\left(i\right)+Q\left(i\right), \end{array}$$
where
  (5) $$\begin{array}{c} P\left(i\right)=\sum_{a\in T_{g}+{\bar{T}}_{g},a>i}\left(a\right), \end{array}$$
  (6) $$\begin{array}{c} Q\left(i\right)=\frac{1}{\sigma_{i}^{j}+2}. \end{array}$$
The individuals having the same raw fitness values are distinguished by calculating their individual density using the K-nearest neighbor method as shown in equation (6). In equation (6), the objective space distance among *i*^th^ and *j*^th^ nearest neighbors is represented by *σ*_*i*_^*j*^ , where $j=\sqrt{A+\bar{A}}$.
Step 3 (selection): this operation copies the nondominated solutions from *T*_g_ and $\bar{T_{g}}$ to ${\bar{T}}_{g+1}$. The following truncation operator is used to reduce ${\bar{T}}_{g+1}$ if its size exceeds the limit of $\bar{A}$:
  (7) i≤ad,a∈T¯g+1⟶:a∈T¯g+1:⇔ 0<j<T¯g+1:σij=σaj∨∃0<j<T¯g+1:∀0<1<j:σil=σal∧σij<σaj.
Else ${\bar{T}}_{g+1}$ is filled with dominated individuals from *T*_*g*_ and $\bar{T_{g}}$. *i* ≤ _*d*_*a* denotes that *i* individual dominates *a* [40].
  Step 4 : in this step, binary tournament selection is implemented by creating a mating pool. In the mating pool, crossover and mutation operations are performed on the individuals selected from ${\bar{T}}_{g+1}$ through tournament selection so that a new population *T*_*g*+1_ is obtained for the next iteration.
  Step 5 : increase *g* as *g*=*g*+1, and if the termination condition *g* ≥ *G* is not satisfied, then go to Step 2; else, represent the archive members as Pareto optimal set [36].

## 4. Performance Analysis

In this paper, MATLAB 2020b online servers with 64-bit, 8-core, and 32 GB RAM are utilized to evaluate the effectiveness of the proposed and the competitive models. The information about the used dataset can be found in [41].

Figure 3 shows the accuracy and loss analysis of the proposed automated diagnosis model. It shows that the proposed diagnosis model achieves significantly better training accuracy and lesser loss value. The proposed model shows a significantly good convergence speed. The proposed model achieves 100% training accuracy during the 150^th^ iteration. The validation accuracy of 99.26% indicates that the proposed model does not suffer from the overfitting issue.

The article "Metaheuristic-based Deep COVID-19 Screening Model from Chest X-Ray Images" was published in 2021. Journal: J Healthc Eng.

Figure 4 shows the confusion matrix analysis of the proposed metaheuristic-based automated diagnosis model. It depicts that the proposed model achieves significantly good accuracy of 98.55%, 100%, 99.2%, and 99.75%, for COVID-19, healthy, pneumonia, and tuberculosis subjects, respectively. Overall, the proposed model achieves 99.5% training accuracy.

Tables 1 and 2 depict the training and validation analysis of the proposed and the existing SPEA-II-based deep transfer learning models on a four-class chest X-ray dataset. The lower difference among Table 1 and 2 values indicates that the SPEA-II-based deep transfer learning models do not suffer much from the overfitting issues. Overall, the proposed model outperforms the competitive SPEA-II-based deep transfer learning models on validation data in terms of accuracy, F-measure, sensitivity, specificity, and area under the curve by 1.23%, 1.18%, 1.26, 1.6%, and 1.13%, respectively.

Table 3 shows the comparison among the existing and proposed SPEA-II-based automated diagnosis models in terms of accuracy. It clearly indicates that the proposed SPEA-II-based automated diagnosis model outperforms the existing models.

## 5. Conclusion

In this paper, a metaheuristic-based deep COVID-19 screening model was proposed for X-ray images. The modified AlexNet architecture was utilized for feature extraction and classification of the input images. Strength Pareto evolutionary algorithm-II (SPEA-II) is used to tune the hyperparameters of modified AlexNet. The proposed model has been tested on a four-class (i.e., COVID-19, tuberculosis, pneumonia, or healthy) dataset. Finally, comparisons were drawn between the existing and the proposed models. Extensive experimental results reveal that the proposed model outperforms the competitive COVID-19 classification models. Overall, the proposed model outperforms the competitive SPEA-II-based deep transfer learning models on validation data in terms of accuracy, *F*-measure, sensitivity, specificity, and area under the curve by 1.23%, 1.18%, 1.26, 1.6%, and 1.13%, respectively. [42]

## Figures and Tables

**Figure 1:** Modified AlexNet Architecture used for COVID-19 classification.

**Figure 2:** *i* ^*th*^ generation of SPEA-II.

**Figure 3:** Accuracy and loss analysis of the proposed COVID-19 classification model.

**Figure 4:** Confusion matrix analysis of the proposed metaheuristic-based deep learning model on a four-class dataset.

**Table 1:** Training analysis of the metaheuristic-based deep learning models.

Models	Accuracy	*F*-measure	Sensitivity	Specificity	Area under the curve
SPEA-II-based VGG19	0.97227	0.97623	0.97565	0.97292	0.97427
SPEA-II-based VGG16	0.99127	0.98302	0.98269	0.99143	0.98709
SPEA-II-based ResNet50	0.98601	0.99151	0.99121	0.98648	0.98880
SPEA-II-based AlexNet	0.99304	0.99660	0.99651	0.99323	0.99484
SPEA-II-based ResNet-34	0.98786	0.99830	0.99824	0.98823	0.99313
SPEA-II-based GoogleNet	0.98952	0.98641	0.98608	0.98977	0.98795
SPEA-II-based InceptionNet	0.99825	0.98981	0.98961	0.99828	0.99397
SPEA-II-based DenseNet201	0.98257	0.98981	0.98947	0.98313	0.98624
SPEA-II-based Xception	0.99475	0.94906	0.94991	0.99466	0.97157
**Proposed SPEA-II-based model**	**0.99976**	**0.99890**	**0.99976**	**0.99890**	**0.99883**

The article "Metaheuristic-based Deep COVID-19 Screening Model from Chest X-Ray Images" was published in 2021. Journal: J Healthc Eng.

**Table 2:** Validation analysis of the metaheuristic-based deep learning models.

Models	Accuracy	*F*-measure	Sensitivity	Specificity	Area under the curve
SPEA-II-based VGG19	0.97735	0.97623	0.97565	0.97789	0.97678
SPEA-II-based VGG16	0.98611	0.98302	0.98269	0.98637	0.98454
SPEA-II-based ResNet50	0.97577	0.99151	0.99121	0.97658	0.98371
SPEA-II-based AlexNet	0.99304	0.99660	0.99651	0.99323	0.99484
SPEA-II-based ResNet-34	0.97923	0.99830	0.99823	0.98843	0.98886
SPEA-II-based GoogleNet	0.98437	0.98641	0.98608	0.98474	0.98540
SPEA-II-based InceptionNet	0.99651	0.98981	0.98961	0.99658	0.99312
SPEA-II-based DenseNet201	0.97409	0.98981	0.98947	0.97491	0.98202
SPEA-II-based Xception	0.98784	0.94906	0.94991	0.98763	0.96824
**Proposed SPEA-II based model**	**0.99130**	**0.99490**	**0.99476**	**0.99154**	**0.99312**

**Table 3:** Accuracy analysis among the proposed SPEA-II-based automated diagnosis model and the existing models.

Model name	Accuracy
CNN [16]	95.3%
MobileNetV2 and SqueezeNet [20]	98.25% and 97.81%
LBP [18]	99%
CNN [17]	97.4%
COVID-Net [19]	92.4%
CovXNet [22]	97.4% for binary and 89.6% for three classes
VGG19 [21]	98.75% for binary and 93.48% for multiclass cases
Xception and ResNet50_V2 [25]	91.4%
ResNet50 [23]	98%
DeTraC [27]	95.12%
Ensemble model [26]	96.4%
Truncated InceptionNet [28]	97.92%
**Proposed model**	**99.13%**

## Data Availability

Data will be made available upon request.
